The article "The Clinical Efficacy of Double Plasma Molecular Absorption System Combined with Plasma Exchange in the Treatment of Acute-on-Chronic Liver Failure: A Systematic Review and Meta-Analysis" was published in 2022. Journal: J Healthc Eng.

# The Clinical Efficacy of Double Plasma Molecular Absorption System Combined with Plasma Exchange in the Treatment of Acute-on-Chronic Liver Failure: A Systematic Review and Meta-Analysis

**DOI:** 10.1155/2022/3139929

**Published:** 2022-03-25

**Authors:** Wenjie Bai, Chun Yao, Dewen Mao, Jinyu Wu, Kejing Wang, Huazhu Wei, Zuhong Huang, Qinglan Shi, Na Wang

**Affiliations:** ^1^Guangxi University of Chinese Medicine, Nanning 530200, China; ^2^The First Affiliated Hospital of Guangxi University of Chinese Medicine, Nanning 530023, China; ^3^Ruikang Hospital Affiliated to Guangxi University of Chinese Medicine, Nanning 530200, China

## Abstract

**Objective:**

This study aims to investigate the clinical efficacy of plasma exchange in treating acute-on-chronic liver failure (ACLF) through meta-analysis.

**Method:**

PubMed, Web of Science, Embase, China National Knowledge Infrastructure (CNKI), and Wanfang databases were searched using a computer for all relevant Chinese and English literature from 2000 to 2021 in each database. At the same time, a large number of related papers and materials were manually consulted. Randomized controlled trials of plasma exchange (PE, control group) and combined double plasma molecular absorption system (DPMAS + PE, observation group) for the treatment of ACLF were collected. Meta-analysis was performed with Stata16.0 software.

**Result:**

A total of 474 articles were retrieved, and 11 papers were finally included for research after screening. Meta-analysis results showed that the effective rate of treatment in the experimental group was significantly higher than that in the control group. At the same time, the observation group's prothrombin activity (PTA) level was better than that of the control group after treatment. After treatment, there was no significant difference in prothrombin time (PT) and international normalized ratio (INR) between the two groups. In addition, after treatment, the alanine aminotransferase (ALT) level of the observation group was significantly lower than that of the control group. However, TBIL levels and albumin (ALB) levels did not change significantly between the two groups. Regarding blood routine indexes, there were no significant changes in creatinine (Cr) levels and platelet counts (PLT) in the two groups after treatment, but hemoglobin (HGB) levels in the observation group were significantly lower than those in the control group.

**Conclusion:**

DPMAS combined with plasma exchange therapy can improve liver function, coagulation function, and blood routine level of ACLF patients and increase the effective rate of treatment. It is an effective treatment for acute-on-chronic liver failure.

The article "The Clinical Efficacy of Double Plasma Molecular Absorption System Combined with Plasma Exchange in the Treatment of Acute-on-Chronic Liver Failure: A Systematic Review and Meta-Analysis" was published in 2022. Journal: J Healthc Eng.

## 1. Introduction

Liver failure is a common clinical syndrome of severe liver disease [1]. Among them, acute-on-chronic liver failure (ACLF) is a common severe acute liver function damage disease, which refers to clinical manifestations of acute (usually within 4 weeks) liver function decompensation on the basis of chronic liver disease, such as coagulopathy, jaundice, hepatic encephalopathy, multiple organ failure, and so on [2]. ACLF is the most common type of liver failure in China. The disease progresses very rapidly. Even after active treatment, the mortality rate is still very high, with a short-term mortality rate of 50% to 90% [3, 4]. Liver transplantation is currently the only effective treatment for ACLF, but due to the lack of a healthy liver source, liver transplantation has not been widely used in clinical practice [5]. Artificial liver support system (ALSS) has become the current first-line clinical treatment method of ACLF due to its ability to restore liver function, improve patient prognosis, and improve patients' quality of life [6–8].

As a commonly used nonbiological artificial liver treatment in clinical practice in China, plasma exchange (PE) uses a membrane plasma separator to separate plasma from whole blood and then replenish the same amount of fresh frozen plasma, which can nonspecifically eliminate liver failure toxins and at the same time supplement essential substances lacking in the patient's body, such as albumin (ALB) and coagulation factors, so as to replace certain functions of the liver [9]. However, there is a severe shortage of blood sources nowadays, and a single replacement with a large amount of fresh frozen plasma will bring risks such as citric acid acidosis, hypocalcemia, allergic reactions, and potential infections. The scope of clinical application is also limited [10, 11]. At present, the double plasma molecular adsorption system (DPMAS) using neutral macroporous resin and ion exchange resin is a new model of the artificial liver [12], which has a better adsorption effect on bilirubin and inflammatory mediators and avoids the risk of blood source tension of plasma exchange, the risks of allergic reactions, and transmitted diseases, and so on and significantly improves the prognosis of patients [13, 14]. However, DPMAS also has shortcomings, such as the inability to supplement albumin, coagulation factors, and other substances and the large loss of albumin and adsorption of coagulation factors [15]. Studies have shown that the two nonbiological artificial liver treatment modes of DPMAS and PE have advantages and disadvantages, which can make up for the shortcomings of separate applications [16]. At present, there are few reports on the use of DPMAS combined with PE for ACLF, and the sample size of individual studies is small, with the results inconsistent between studies. There is still a lack of systematic reviews on the effectiveness of DPMAS combined with low-volume PE in the treatment of acute-on-chronic liver failure. This study aims to systematically evaluate existing randomized controlled trials (RCT) studies through meta-analysis and provide evidence-based medical evidence for the further clinical use of DPMAS combined with PE in the treatment of ACLF.

The article "The Clinical Efficacy of Double Plasma Molecular Absorption System Combined with Plasma Exchange in the Treatment of Acute-on-Chronic Liver Failure: A Systematic Review and Meta-Analysis" was published in 2022. Journal: J Healthc Eng.

## 2. Materials and Methods

### 2.1. Literature Search

Literature searches were conducted through PubMed, Web of Science, Embase, CNKI, and Wanfang databases for literature retrieval with the time set from 2010 to 2021. The search terms used for both languages (Chinese and English) were: (1) “plasma exchange,” (2) “chronic and acute,” (3) “liver failure,” and (4) “clinical efficacy.”

### 2.2. Inclusion and Exclusion Standards

#### 2.2.1. Inclusion Criteria

Inclusion criteria of the study were as follows: (1) population: patients diagnosed with ACLF; (2) intervention: o the basis of conventional treatment, patients in the observation group were treated with a double plasma molecular absorption system combined with plasma exchange (DPMAS + PE); (3) comparison group: patients were treated with only plasma exchange therapy (PE); (4) outcomes: treatment effective rate, after treatment prothrombin activity (PTA), prothrombin time (PT), international normalized ratio (INR), total bilirubin (Tbil), alanine aminotransferase (ALT), albumin (ALB), creatinine (Cr), platelet count (PLT), hemoglobin (HGB), and any other indicators; and (5) study: RCT.

#### 2.2.2. Exclusion Criteria

Exclusion criteria of the study were as follows: (1) overview, adverse reaction reports, and nonclinical trial studies such as pharmacology and pharmacokinetics; (2) unable to obtain original literature materials and data; and (3) repeated literature publications.

### 2.3. Data Extraction and Analysis

Relevant data were extracted to EndNote 7.0 and collated. Two reviewers independently screened the literature according to the inclusion and exclusion criteria and extracted and sorted the data. By reviewing the title, content, research methods, and abstracts of the literature, the literature consistent with this research was selected. Disagreements were resolved through discussion or negotiation with a third evaluator. Authors were contacted to consult data metrics not mentioned in the literature if necessary. The main contents of data extraction include (1) basic information in the literature, (2) types of research methods, (3) sample size, and (4) outcome indicators.

The article "The Clinical Efficacy of Double Plasma Molecular Absorption System Combined with Plasma Exchange in the Treatment of Acute-on-Chronic Liver Failure: A Systematic Review and Meta-Analysis" was published in 2022. Journal: J Healthc Eng.

### 2.4. Statistical Analysis

All statistical analyses were performed using Stata 16.0 software (StataCrop, Texas, USA). First, the *χ*^2^ test was used to test the heterogeneity of the results of each study, and the test level was *α* = 0.05. If I^2^ > 50% and *P* < 0.05, statistical heterogeneity was assessed as high. And the random-effects model was used for the meta-analysis. Otherwise, the fixed-effects model was employed. When the number of studies exceeds 5, a funnel chart was used to analyze the bias of the studies. The measurement data used the standardized mean difference (SMD) as the measurement index, and the categorical variables used the odds ratio (OR) and the 95% confidence interval (CI) as the measurement indexes. When *P* < 0.05, the difference was statistically significant.

## 3. Results

### 3.1. Search Results

A total of 474 documents were retrieved according to the search strategy, of which 179 duplicate articles were excluded, 76 articles marked as unqualified by automated tools were eliminated, and 92 cases were excluded through title/abstract inspection. Through the further reading of the full text, 116 articles that did not meet the criteria were excluded, and 11 studies were finally included [12, 15, 17–25]. The literature screening process was shown in Figure 1. The characteristics of each included study are shown in Table 1, which summarized the detailed information of the included study design, participants, intervention measures, and results.

### 3.2. Comparison of Treatment Efficiency

Eleven studies [12, 15, 17–25] reported on the effective rate of treatment. The included studies were tested for heterogeneity (*I*^2^ = 0.0%, *P* = 0.782), indicating no heterogeneity among the included studies, and the fixed-effect model was used to combine effect size. Meta-analysis results showed that the effective rate of treatment in the experimental group was significantly higher than that in the control group (OR = 1.739, 95% CI (1.279, 2.365), *P* < 0.001; Figure 2(a)). Sensitivity analysis results showed (Figure 2(b)) that Xie et al. [15] might affect the heterogeneity through elimination method one by one, but the results obtained still suggested that the experimental group had higher effective rates than the control group. Therefore, the results of this study were relatively stable and reliable. In addition, Begg's funnel plot (Figure 2(c)) did not show significant asymmetry in the overall meta-analysis of publication bias.

### 3.3. Comparison of Coagulation Function after Treatment

There were seven studies [12, 15, 18–20, 22, 25] that reported the effect of DPMAS combined with PE on the PTA level of ACLF patients. The included studies have significant heterogeneity (I^2^ = 93.6%, *P* ≤ 0.001), and a random-effects model was employed. The results showed that the PTA level of the experimental group was significantly higher than that of the control group (SMD = 1.239, 95% CI (0.513, 1.966), *P* = 0.001; Figure 3(a)).

The article "The Clinical Efficacy of Double Plasma Molecular Absorption System Combined with Plasma Exchange in the Treatment of Acute-on-Chronic Liver Failure: A Systematic Review and Meta-Analysis" was published in 2022. Journal: J Healthc Eng.

Five studies [12, 15, 18, 21, 24] reported the INR level after treatment. Similarly, there were also five studies [15, 17–19, 23] reporting the level of PT after treatment. There was significant heterogeneity in the included studies (INR: *I*^2^ = 82.6%, *P* ≤ 0.001; PT: *I*^2^ = 86.7%, *P* ≤ 0.001), and the random-effects model was used to combine the effect sizes. The results showed no significant difference in INR and PT levels between the two groups of patients after treatment (*P* = 0.575 and *P* = 0.451; Figures 3(b) and 3(c)).

Due to the heterogeneity among the included studies, sensitivity analysis was required. Through the one-by-one elimination method, it is found that Li et al. [19], Yao et al. [12], and Chen et al. [23] were the main sources of heterogeneity increase of PTA, INR, and PT, respectively. After excluding these three articles, the results obtained still showed no significant difference (Figure 4(a)–4(c)). Therefore, the results of this study were relatively stable and reliable.

### 3.4. Comparison of Liver Function after Treatment

Eleven studies [12, 15, 17–25] reported the effect of DPMAS combined with PE treatment on the TBIL levels in ACLF patients. A heterogeneity test was performed on the included studies (*I*^2^ = 36.7%, *P* = 0.106), indicating that there was no heterogeneity among the included studies, and a fixed-effects model was used for the meta-analysis. The results showed that there was no significant difference in TBIL levels between the two groups of patients after treatment (SMD = −0.392, 95% CI (−0.531, 0.253), *P* < 0.001; Figure 5(a)).

Eight studies [15, 17, 18, 20–22, 24, 25] reported the effect of DPMAS combined with PE treatment on ALT levels in ACLF patients, and nine studies [12, 15, 17–19, 21–24] reported the effect on ALB levels. The included studies have significant heterogeneity (ALT: *I*^2^ = 69.1%, *P* = 0.002; ALB: *I*^2^ = 93.9%, *P* ≤ 0.001), and the random-effects model was used for analysis. The results showed that the ALT level of the observation group was superior to that of the control group (SMD = −0.517, 95% CI (−0.820, −0.214), *P* = 0.001), while the ALB level had no significant difference between the two groups (SMD = 0.206, 95% CI (−0.445, 0.857), *P* = 0.535; Figures 5(b) and 5(c)).

Sensitivity analysis results showed that through the one-by-one elimination method, it was found that Xie et al. [15] might affect the heterogeneity of the study on TBIL levels, and the statistical results of the effective value of this study were stable after the elimination (Figure 6(a)). Due to the heterogeneity between the included studies of ALT level and ALB level, by eliminating one by one, it was found that Qin and Wei 2019 [22] and Liu et al. [17] might be the main source of heterogeneity in ALT and ALB elevation. After excluding these two articles, the results obtained were still similar to the previous ones (Figures 6(b) and 6(c)). Therefore, the results of this study were relatively stable and reliable.

The article "The Clinical Efficacy of Double Plasma Molecular Absorption System Combined with Plasma Exchange in the Treatment of Acute-on-Chronic Liver Failure: A Systematic Review and Meta-Analysis" was published in 2022. Journal: J Healthc Eng.

### 3.5. Comparison of Routine Blood Levels after Treatment

Five studies [12, 15, 18–20] reported the effect of DPMAS combined with PE treatment on Cr levels in patients with acute-on-chronic liver failure. Six studies [15, 17, 19, 20, 22] reported changes in PLT levels after treatment, and four studies [15, 17, 19, 20] reported changes in HGB levels after treatment. The included studies were tested for heterogeneity (Cr: *I*^2^ = 0.0%, *P* = 0.998; PLT: *I*^2^ = 31.3%, *P* = 0.201; HGB: *I*^2^ = 0.0%, *P* = 0.579), indicating that there was no heterogeneity among the included studies, and the fixed-effects model was used. The results showed that there was no significant difference in Cr levels (SMD = −0.065, 95% CI (−0.256, 0.126), *P* = 0.506) and PLT levels between the two groups after treatment (SMD = −0.173, 95% CI (−0.361, 0.016), *P* = 0.073). However, the HGB level of the observation group was significantly lower than that of the control group (SMD = −0.256, 95% CI (−0.490, −0.022), *P* = 0.032; Figures 7(a)–7(c)). The sensitivity analysis results showed that the research reports were eliminated one by one. The results showed that the pooled effect size was still statistically arguable, and the forest plot direction did not change significantly before and after the elimination (Figures 8(a)–8(c)).

## 4. Discussion

ACLF is a major critical complication in patients with liver disease. More than 80% of ACLF is caused by acute exacerbations of chronic hepatitis B caused by hepatitis B virus infection. ACLF has a complex etiology and can present clinically as systemic infection, systemic jaundice, and coagulation dysfunction until systemic multiple organ failure with a relatively high short-term mortality rate [26–28]. In the introduction, we have summarized the effects of DPMAS or PE alone and combined DPMAS on the clinical efficacy of ACLF patients. To further clarify the clinical efficacy differences between the two treatment methods, this study explores the difference in the clinical efficacy of the two treatments methods: DPMAS combined with PE and PE alone in ACLF patients.

The article "The Clinical Efficacy of Double Plasma Molecular Absorption System Combined with Plasma Exchange in the Treatment of Acute-on-Chronic Liver Failure: A Systematic Review and Meta-Analysis" was published in 2022. Journal: J Healthc Eng.

The liver clearance function of ACLF patients was significantly reduced. A large amount of endogenous toxic substances accumulated in the patient's body, such as various water-soluble toxin, protein-bound toxins, and metabolites, which seriously affect hepatocyte regeneration and the recovery of liver function in ACLF patients. ACLF can also affect other vital organs, causing multiple organ dysfunction, high mortality rates, and an extremely poor prognosis [29, 30]. Although PE cannot directly improve the synthesis and detoxification functions of the liver, it can remove small- and medium-sized metabolic toxins, proteins, immune complexes, and other macromolecular substances in the body. At the same time, it can supplement the essential substances lacking in the body, such as albumin and coagulation factors [31]. Therefore, it can replace certain functions of the liver [32]. Larsen et al. [33] showed that high-dose PE could significantly improve the prognosis of patients with acute liver failure, improve the clinical treatment outcomes, and improve the quality of life. Studies have also shown that PE can improve the liver function and prognosis of patients with acute-on-chronic liver failure to a certain extent [34]. This study found that DPMAS combined with PE treatment and PE treatment alone can both effectively reduce ALT, ALB, and TBIL levels in ACLF patients, which is consistent with the results of previous studies. In addition, the ALT level of patients in the DPMAS combined PE treatment group was better than that of the PE alone treatment group. This may be because DPMAS uses two adsorption columns of neutral macroporous adsorption resin and ion exchange resin to continuously adsorb plasma and then returns it to the body. It provides an effective method to continuously remove macromolecules in plasma and endogenous toxic substances bound to proteins from plasma and at the same time specifically remove bilirubin, without the need for plasma supplementation or fluid replacement during treatment [12].

Studies have found that DPMAS can better remove bilirubin, but it may reduce some of the beneficial components in the blood, such as the appearance of ALB decline and PT prolongation, which may be related to the nonselective adsorption of a small amount of albumin and coagulation factors in the blood by the adsorption column [35]. Studies have shown that DPMAS combined with PE can supplement a certain amount of plasma to improve the coagulation function while actively supplementing albumin to reduce hypoproteinemia, effectively avoiding bleeding risks and hypoalbuminemia. This study found that after DPMAS combined with PE and PE alone treatment, the patient's PTA levels were significantly increased with better results in the DPMAS combined with PE treatment group than PE treatment alone. While both INR and PT levels decreased, there was no significant difference between the two groups. In addition, the HGB and PLT of the two groups of patients decreased. The level of HGB in the DPMAS + PE treatment group was superior to PE treatment alone, which may be related to the adsorption material used and the membrane biocompatibility of the plasma separator used or may be associated with the destruction of red blood cells and platelets due to the mechanical loss of blood in the extracorporeal circulation during the treatment procedure [15]. Still, no serious adverse events such as obvious bleeding, hemolysis, and so on occurred. DPMAS + PE treatment and PE treatment alone had no significant effect on the Cr levels of patients, suggesting good safety, which is consistent with the results of previous studies [36].

The article "The Clinical Efficacy of Double Plasma Molecular Absorption System Combined with Plasma Exchange in the Treatment of Acute-on-Chronic Liver Failure: A Systematic Review and Meta-Analysis" was published in 2022. Journal: J Healthc Eng.

However, in general, this study has some limitations. (1) This study mainly collects relevant literature by searching electronic databases and manual screening of included literature and references. Missed detection was caused by possible shortcomings in the included literature and search strategy in the electronic database. (2) Eleven included literature inevitably had certain heterogeneity due to different selection of drugs and dosage, frequency, and course of treatment in the control and experimental groups. (3) Only one of eleven included study designs was an international study, and the rest were all selected domestic studies. Based on clinical randomized controlled trials, the quality of the comprehensive evaluation literature was not very high, and the statistical results may be biased. Therefore, large-sample, high-quality, multicenter randomized controlled clinical trials need to be carried out to enhance the accuracy and credibility of the research results in order to provide more efficient methods for the next clinical treatment step.

## 5. Conclusion

In summary, DPMAS combined with PE therapy can improve the effectiveness of ACLF therapy, effectively protect patients' liver function and blood coagulation function, maintain blood routine levels, and improve its clinical efficacy.

## Figures and Tables

**Figure 1:** Literature screening flow chart.

**Figure 2:** A meta-analysis of the effective rate of DPMAS combined with PE in the treatment of patients with acute-on-chronic liver failure: (a) forest plot comparing the effective rate of PE and DPMAS in the treatment of patients with acute-on-chronic liver failure, (b) sensitivity analysis of effective rate, and (c) funnel plot assessing potential publication bias in effective rate studies. PE: plasma exchange and DPMAS: double plasma molecular absorption system.

The article "The Clinical Efficacy of Double Plasma Molecular Absorption System Combined with Plasma Exchange in the Treatment of Acute-on-Chronic Liver Failure: A Systematic Review and Meta-Analysis" was published in 2022. Journal: J Healthc Eng.

**Figure 3:** The forest plot analysis of coagulation function in patients with acute-on-chronic liver failure treated by DPMAS combined with PE. Forest plot comparing the prothrombin activity after treatment (PTA) level (a), international normalized ratio after treatment (INR) level (b), and prothrombin time (PT) level (c) in the coagulation function of patients with acute-on-chronic liver failure treated with DPMAS combined with PE.

**Figure 4:** Sensitivity analysis of coagulation function in patients with acute-on-chronic liver failure treated with DPMAS combined with PE: (a) sensitivity analysis of PTA levels, (b) sensitivity analysis of INR levels, and (c) sensitivity analysis of PT levels.

**Figure 5:** The forest plot analysis of liver function in patients with acute-on-chronic liver failure treated by DPMAS combined with PE. Forest plot comparing the liver function total bilirubin (TBIL) levels (a), alanine aminotransferase (ALT) levels (b), and albumin (ALB) levels (c) of patients with acute-on-chronic liver failure treated with DPMAS combined with PE.

**Figure 6:** Sensitivity analysis of liver function in patients with acute-on-chronic liver failure treated by DPMAS combined with PE: (a) sensitivity analysis of TBIL levels, (b) sensitivity analysis of ALT levels, and (c) sensitivity analysis of ALB levels.

**Figure 7:** Forest plot analysis of blood routine in patients with acute-on-chronic liver failure treated with DPMAS combined with PE. Forest plot compares the changes of creatinine (Cr) levels (a), platelet count (PLT) levels (b), and hemoglobin (HGB) levels (c) in patients with acute-on-chronic liver failure patients treated with DPMAS combined with PE.

**Figure 8:** Sensitivity analysis of blood routine in patients with acute-on-chronic liver failure patients treated with DPMAS combined with PE: (a) Cr level sensitivity analysis, (b) PLT level sensitivity analysis, and (c) HGB level sensitivity analysis.

**Table 1:** Basic characteristics of the included literature.

Study	Year	Sample time (year.month)	Cases treat/con	Age (years)		Sex (male/female)		Study design	Outcome measures
				Treat group	Treat group	Treat group	Con group		
Liu Xiaoyan	2018	2016.02∼2016.12	30/32	45 ± 12	42 ± 13	26/4	28/4	Retrospective	①④⑤⑥⑦⑨⑩

Du Zhen	2021	2016.06∼2018.12	34/38	47.5 ± 10.2	48.2 ± 8.5	28/6	29/9	Retrospective	①②③④⑤⑥⑦⑧

Li Yongchao	2020	2016.09∼2017.10	30/30	42.1 ± 2.3	42.1 ± 2.3	17/13	17/13	RCT	①②⑤⑦⑧⑨⑩

Zuo Tongkun	2020	2013.01∼2019.01	25/25	46.25 ± 12.05	43.68 ± 11.87	19/6	18/7	Retrospective	①②⑤⑥⑧⑨⑩

Li Chunyu	2021	NR	35/32	49.12 ± 6.54	49.31 ± 5.98	21/14	20/12	RCT	①③④⑤⑥⑦

Qin Hua	2019	2016.1∼2018.12	32/37	45.1 ± 10.6	42.8 ± 11.3	26/6	29/8	Retrospective	①②⑤⑥⑦⑨

Xie Nengwen	2021	2018.01∼2019.12	56/56	36.30 ± 5.41	35.89 ± 4.88	38/18	40/16	Retrospective	①②③④⑤⑥⑦⑧⑨⑩

Chen Li	2020	2013.01∼2019.06	30/23	49.3 ± 12.08	46.7 ± 10.9	20/10	20/3	Retrospective	①④⑤⑦

Jia Yao	2019	2016.06∼2018.06	54/77	47.6 ± 11.5	43.8 ± 14.2	38/16	54/23	Retrospective	①②③⑤⑦⑧

Nong Cunli	2019	2015.01∼2017.12	33/31	39.33 ± 8.16	39.26 ± 9.27	28/5	27/4	RCT	①③⑤⑥⑦

Qin Hao	2020	2017.01∼2018.12	43/43	45.63 ± 5.51	45.16 ± 5.47	24/19	25/18	RCT	① ②⑤⑥⑨

*Note.* Treat: treatment; Con: control; RCT: randomized controlled trial; and NR: not reported. ① effective rate, ② prothrombin activity after treatment (PTA), ③ international normalized ratio after treatment (INR), ④ prothrombin time after treatment (PT), ⑤ total bilirubin level after treatment (TBIL), ⑥ alanine aminotransferase level after treatment (ALT), ⑦ albumin level after treatment (ALB), ⑧ creatinine level after treatment (Cr), ⑨ platelet level after treatment (PLT), and ⑩ hemoglobin level after treatment (HGB).

The article "The Clinical Efficacy of Double Plasma Molecular Absorption System Combined with Plasma Exchange in the Treatment of Acute-on-Chronic Liver Failure: A Systematic Review and Meta-Analysis" was published in 2022. Journal: J Healthc Eng.

## Data Availability

The data used to support the findings of this study are available from the corresponding author upon request.
